# Legal Text Recognition Using LSTM-CRF Deep Learning Model

This article has been retracted.

**DOI:** 10.1155/2022/9933929

**Published:** 2022-03-17

**Authors:** Hesheng Xu, Bin Hu

**Affiliations:** Department of Law, Zhejiang University City College, Hangzhou 310015, China

## Abstract

In legal texts, named entity recognition (NER) is researched using deep learning models. First, the bidirectional (Bi)-long short-term memory (LSTM)-conditional random field (CRF) model for studying NER in legal texts is established. Second, different annotation methods are used to compare and analyze the entity recognition effect of the Bi-LSTM-CRF model. Finally, other objective loss functions are set to compare and analyze the entity recognition effect of the Bi-LSTM-CRF model. The research results show that the F1 value of the model trained on the word sequence labeling corpus on the named entity is 88.13%, higher than that of the word sequence labeling corpus. For the two types of entities, place names and organization names, the F1 values obtained by the Bi-LSTM-CRF model using word segmentation are 67.60% and 89.45%, respectively, higher than the F1 values obtained by the model using character segmentation. Therefore, the Bi-LSTM-CRF model using word segmentation is more suitable for recognizing extended entities. The parameter learning result using log-likelihood is better than that using the maximum interval criterion, and it is ideal for the Bi-LSTM-CRF model. This method provides ideas for the research of legal text recognition and has a particular value.

## 1. Introduction

In the 21st century, the rapid development of science and technology, the era of artificial intelligence (AI), and cloud computing have come one after another. As the carrier of network interconnection, the computing power of computers has been dramatically improved. As an algorithm that has emerged in recent years, deep learning has been widely used in the Internet, transportation, medical care, construction, and other fields [1]. Since named entity recognition (NER) was proposed, the categories of named entities have been continuously expanded and improved. With the development of AI technology, time and labor costs have significantly reduced the recognition of NER [2]. The research fields of named entities include journalism, biology, medicine. Each domain has its characteristics. In the legal area, the identification of named entities in legal texts can be extracted from the text [3].

The research fields of named entities include journalism, biology, medicine, and other areas. Different fields have their characteristics. In the legal field, legal texts are identified by named entities. Entities with specific meanings extracted from legal texts help judicial practitioners to improve decision-making efficiency. In 2013, China Judgements Online began to publish effective judgment documents. As of March 9, 2021, the total number of effective judgment documents announced has exceeded 110 million. This provides data support for NER research in the legal field. Correctly identifying legal entities in judicial documents is the basis for subsequent processing tasks, such as event extraction and relationship extraction. Therefore, in response to the actual needs in the judicial field, the research on the NER method of Chinese legal texts has become essential [4]. Traditional machine learning requires the statistics and analysis of readers to dig out features that impact the task. With the development of computer technology, neural network models have been used in various natural language processing tasks in recent years. The neural network model does not depend on feature engineering, saving time and labor costs. The expression of word vectors has brought a powerful development momentum to the development of named entities. The representation of word vectors can represent more semantic information than manually extracted features, and the model that enables word vectors to obtain more semantic information is constantly updated.

The Bi-LSTM model and CRF model are commonly used models for NER. The Bi-LSTM model avoids the problem of long-term dependence, enables the model to learn more distant information, and gives it the ability to obtain contextual information. The CRF model not only uses internal information but also uses contextual information to mark a location. The Bi-LSTM-CRF model combines the advantages of the two models and is also a mainstream model for NER. The innovation is to establish the Bi-LSTM-CRF model, set different target loss functions, and use different labeling methods to compare and analyze the established model's legal text entity recognition effect. This study can make up for the deficiencies in the research of legal text recognition, reduce the workload of judicial personnel, and effectively improve the efficiency of judicial case acceptance, registration, and review.

## 2. Literature Review

For different fields, entity recognition research will be additional. Zhang et al. [5] proposed a Chinese character-based enhancement NER model. It aimed at the problems of Chinese NER in apple diseases and insect pests, including many types of entities, entities with aliases or abbreviations, and difficulties in identifying rare entities. Deep learning has produced the most advanced performance on many natural language processing tasks, including NER. Liu et al. [6] proposed a hybrid deep learning method in the medical field to improve the recognition accuracy of NER. Specifically, a two-way encoder representation model is used to extract the basic features of the text. Long and short-term memory (LSTM) learns the representation of the text context and combines the mechanism of multihead attention to extracting chapter-level features. Identifying uncommon or emerging named entities in the user-generated text is challenging, especially when using informal or slang text. Al-Nabki et al. [7] solved this shortcoming by proposing local distance neighbors. Local distance neighbors are a new feature that replaces place-name indexing. This method allows the model to obtain the most advanced results. Affi et al. [8] introduced a deep neural network (DNN) model to solve a challenging task of sequence labeling problem, the NER task. Carbonell et al. [9] introduced a lightweight architecture for NER. The model consists of a convolutional character, word encoder, and an LSTM tag decoder. It is based on the task standard. Nearly, state-of-the-art performance is achieved on the data set, and the computational efficiency is much higher than the best-performing model. In recent years, the development of DNN and the advancement of pretrained word embedding have become the driving force of neural networks. In this case, making full use of the information extracted from embedded terms requires more in-depth research. Wang et al. [10] proposed an adversarial training system, which improved the existing NER method from two aspects: model structure and training process. In addition, it also presented a unique harmful training method. The training method solves the problem of overfitting in the network. During the training process, the variables are more diversified by adding disturbance to the variables in the network. Thereby, it improves the generalization and robustness of the model. Text features can be obtained with the in-depth study of text features. But in the judicial field, there is not much research on identifying legal texts.

The rule-based method requires manual construction of rule templates, which is too costly and has certain limitations. Statistical machine learning methods are used for NER models: maximum entropy, support vector machine, and conditional random field. With the maturity of electronic hardware and the emergence of word vectors, deep learning can be trained on the large-scale corpus. Nowadays, many NER methods based on deep understanding have achieved good results. The work in the legal field mainly includes text classification, prediction of judgment results, and information extraction of entities in the text. Because of the lack of annotated corpus of early legal texts and the more incredible difficulty of entity recognition in Chinese texts, the research on NER of legal texts cannot achieve good results. Nowadays, new models and optimization methods are proposed, making it possible to identify named entities from legal texts better.

## 3. Materials and Methods

### 3.1. NER

Named entities refer to those words or phrases that contain special meaning or strong references [11]. Under normal circumstances, the entity types include some names, place names, and organization names. For example, “Shanghai” and “Zhejiang” are all name entities. But there will also be some specific entity types appearing in particular fields, such as medical treatment and law [12]. NER refers to the classification of named entities. Of course, the classification process is completed on the computer. The main goal of NER is to extract some essential information from the text. The accuracy of the key information extraction will directly affect the next task [13, 14]. The NER task must generally meet three measurement criteria to be recognized as correct. The specific criteria are shown in Figure 1.

Under normal circumstances, the recognition of each type of entity by NER can be regarded as a binary classification problem, so the accuracy rate, recall rate, and F1 value can be used to evaluate the model. But before calculating these three indicators, it is necessary to make summary statistics on the predicted category and the correct category of the entity separately [15]. Taking the recognition of place names by the model as an example, the calculation equations of these three indicators are expressed. Suppose that the number predicted by the model and the actual entity is the place's name is marked as TP. The number indicated by the model is marked, and the fact that the entity is not a name named TN. The number of predicted entities is marked with place names that are not place names as FP. The number of predicted entities that are not place names is marked but place names as FN. Then, precision, recall, and F1-score are represented by (1), (2), and (3), respectively:

(1) $$\begin{array}{c} \text{precision}=\frac{\text{TP}}{\text{TP}+\text{FP}}, \end{array}$$

(2) $$\begin{array}{c} \text{recall}=\frac{\text{TP}}{\text{TP}+\text{FN}}, \end{array}$$

(3) $$\begin{array}{c} F1-\text{score}=2\times \frac{\text{precision}\times \text{recall}}{\text{precision}+\text{recall}}. \end{array}$$

### 3.2. Annotation Coding Method

NER using deep learning needs to use word vectors, and its premise is to segment the text. A good word segmentation can make correct segmentation of ambiguous sentences and must have good segmentation details. This paper compares the word segmentation effect of commonly used word segmentation tools and chooses a word segmentation tool suitable for the Chinese word segmentation system. This word segmentation tool can significantly impact Chinese legal texts' word segmentation and affinity. The person's name is recorded as PER, the place's name is registered as LOC, and the organization's name is recorded as ORG. The names of persons, businesses, and organizations are identified in the legal text. The {PER, ORG, LOC} in the entity label corresponds to {person name, organization name, place name}, and the BIO labeling method is combined with the entity's {PER, ORG, LOC} labeling method. For example, B-PER means the beginning of the named entity, I-PER means the middle or end, and O means nonentity. Combining the Begin-Inside-Outside (BIO) labeling method with the entity labeling method, the specific representation is shown in Table 1.

### 3.3. Long Short-Term Memory (LSTM) Network

Deep learning has a strong ability to learn characteristics and analyze rules between data. This technology is conducive to the promotion of data visualization and the development of classified management data. The working principle of deep learning is to gradually approximate complex functions by learning from deep nonlinear networks [16]. Compared with traditional artificial neural networks, deep learning model structure learning is more in-depth. There are many nodes in the hidden layer, emphasizing the feature learning of the data [17]. Deep learning converts the feature representation of samples in the original space into a new feature space, simplifying data classification and prediction. Deep learning learns from fewer samples and expresses complex functions with fewer parameters, which reduces the difficulty of setting and adjusting model parameters. Deep learning contains more hidden layers than traditional shallow neural networks, with richer sample features that can be learned and better simulation performance [18].

LSTM is essentially derived from the recurrent neural network (RNN) [19]. RNN is an extraordinary network for processing serial data. Its most significant advantage is that it has a memory function and solves current output and previous input problems. For example, when processing a piece of text information, the received information can be understood with the help of prior memory. In general, RNN is not limited by the length of the data sequence to be processed and can quickly and accurately analyze data sequences of any size [20]. However, model training is not easy to implement in practical applications, and even the previous memory disappears. The main reason for this situation is that RNN will produce gradient disappearance when reverse derivation of long sequence data. LSTM was proposed to solve the shortcomings of RNN [21, 22].

LSTM is adding a state unit to the RNN. The function of LSTM is to save previously entered information. In general, the tanh function is selected as the activation function of the input and output of the memory unit, and the sigmoid function is used as the activation function of the gate structure [23, 24]. The output value of the sigmoid function is between (0, 1), as shown in equation (4) as follows:

(4) $$\begin{array}{c} \text{sigmoid}\left(x\right)=\frac{1}{1+e^{-x}}. \end{array}$$

The output value of the tanh function is between (−1, 1), as shown in (5) as follows:

(5) $$\begin{array}{c} \text{tan}h\left(x\right)=\frac{1-e^{-2x}}{1+e^{-2x}}. \end{array}$$

The structure of LSTM is shown in Figure 2.

The specific algorithm is as follows:

(1) Forget door: effectively judge whether the information in the storage unit is retained or not, the input information and the hidden state of the previous point in time will have a particular impact on the forget gate [25]. The specific calculation is shown in
  (6) $$\begin{array}{c} f_{t}=\text{sigmoid}\left(U_{f}x_{t}+W_{f}h_{t-1}+b_{f}\right), \end{array}$$
*U*_*f*_ is the weight matrix connected with the input data, *b*_*f*_ is the bias vector, and *W*_*f*_ is the weight matrix connected with the previously hidden layer.
(2) Input gate: the input gate is to control the data to be updated. Like the forget gate, it is affected by the input information and the hidden state at the previous time. The specific calculation is shown in
  (7) $$\begin{array}{c} i_{t}=\text{sigmoid}\left(U_{i}x_{t}+W_{i}h_{t-1}+b_{i}\right), \end{array}$$
*U*_*i*_ is the weight matrix connected with the input data, *b*_*i*_ is the bias vector, and *W*_*i*_ is the weight matrix connected with the previously hidden layer.
(3) Memory information: the memory information is on the latest input data, and the value to be added to the memory module is calculated. Its influencing factors are the same as the forget gate and output gate [26]. The specific calculation is shown in
  (8) $$\begin{array}{c} a_{t}=\tanh\left(U_{a}x_{t}+W_{a}h_{t-1}+b_{a}\right), \end{array}$$
*U*_*a*_ is the weight matrix connected to the input data in the memory information, *b*_*a*_ is the bias vector, and *W*_*a*_ is the weight matrix connected to the previously hidden layer in the memory information.
(4) Cell unit: its function is to update the state value of the memory unit in the storage module. The specific calculation is shown in
  (9) $$\begin{array}{c} C_{t}=C_{t-1}\cdot f_{t}+i_{t}\cdot a_{t}+b_{i}, \end{array}$$
*C*_*t*−1_ is the state value corresponding to the memory unit at the previous time node, *f*_*t*_ and *i*_*t*_ are the calculated values of the forget gate and the input gate, respectively, and *a*_*t*_ is the value corresponding to the memory information waiting to be updated.
(5) Output gate: the output gate is to controls the output of the entire network. Its influencing factors are also the same as the influencing factors of the input gate. The specific calculation is shown in
  (10) $$\begin{array}{c} o_{t}=\text{sigmoid}\left(U_{o}x_{t}+W_{o}h_{t-1}+b_{o}\right). \end{array}$$
*U*_*o*_ is the weight matrix connected to the input data in the output gate, *b*_*o*_ is the bias vector, and *W*_*o*_ is the weight matrix connected to the previously hidden layer in the output gate.
(6) Network output value: the network output value is the calculation of the final output in the network. The specific calculation is shown in
  (11) $$\begin{array}{c} h_{t}=o_{t}\cdot \;\tanh\left(C_{t}\right). \end{array}$$

*o*_*t*_ is the value of the output gate, and *C*_*t*_ is the state value of the cell unit.

The training process of the LSTM network is the same as the training process of other neural networks. Both include forward and backward propagation methods. The specific training steps are shown in Figure 3. However, the more popular two-way LSTM model is used here, expressed as bidirectional LSTM (Bi-LSTM).

### 3.4. Conditional Random Fields (CRFs)

CRF is a conditional probability distribution model of another set of output sequences under the condition of a group of known input sequences. CRF has been widely used in natural language processing. CRF can provide certain constraints on the label to ensure that the output label is within a reasonable range [27, 28]. Suppose that *Y*={*Y*_*v*_*|v* ∈ *V*}, *V* and *E* represent the set of nodes and edges, respectively, and there is an undirected graph *G*=(*V*, *E*) composed of *Y*. Use it to describe the Markov random field, which can be expressed as

(12) $$\begin{array}{c} P\left(Y_{v}|X,Y_{w},w\neq v\right)=P\left(Y_{v}|X,Y_{w},w:v\right). \end{array}$$

*Y*_*v*_ is the random variable corresponding to node *v*, and *X* is the observation sequence. *w* ≠ *v* is all the remaining nodes except node *v*, *Y*_*w*_ is the random variable corresponding to node *w*, and *w* ~ *v* is all nodes *w* connected to the edges of node *v* in the undirected graph. In general, the CRF model is modelled according to the conditional probability distribution *P*(*Y|X*), which is an orderly solution to the probability distribution of *Y* under the condition of *X*. The steps to solve the sequence labeling problem through the CRF model are as follows:

Suppose there is an input sequence of length *n* as *X*, expressed as

(13) $$\begin{array}{c} X=\left(x_{1},x_{2}\ldots ,x_{n}\right). \end{array}$$

Then, the label sequence *Y* at this time is expressed as

(14) $$\begin{array}{c} Y=\left(y_{1},y_{2}\ldots ,y_{n}\right). \end{array}$$

The CRF model is used to calculate the sentence, and the calculated result includes two parts, the score of the letter mark and the mark after the transfer. The score of the letter mark is a matrix, and the score of the impact after the transfer is the modulus parameter. The specific calculation of the final score *P* is shown in

(15) $$\begin{array}{c} P=\sigma \left(V\left[x_{1},x_{2},\ldots ,x_{n}\right]+d\right). \end{array}$$

*V* is the weight parameter, *d* is the bias term, *k* is the number of marked categories, and *σ*(*·*) is the activation function.

Through the calculation of the above equation, the score of the prediction result sequence can be obtained, which can be expressed as

(16) $$\begin{array}{c} S=\left(X,y,\theta \right)=\sum_{i=0}^{n}A_{y_{i},y_{i+1}}+\sum_{i=1}^{n}P_{i,y_{i}}. \end{array}$$

A is the score matrix of the transfer of the marker, its size is (*k*+2)*∗*(*k*+2), *θ* is the model parameter, and *A*_*i*,*j*_ is the score of the marker *j* connected to the marker *i*.

The calculated prediction results are screened, and the score of the appropriate prediction result sequence is calculated. Under the premise of the existence of sequence *X*, the probability of occurrence of the prediction result sequence *y* is solved, and the specific calculation is expressed as shown in

(17) $$\begin{array}{c} P\left(y|X,\theta \right)=\frac{e^{s\left(X,y,\theta \right)}}{\sum {}_{\tilde{y}\in Y_{X}}e^{s\left(X,\tilde{y},\theta \right)}}. \end{array}$$

*Y*_*X*_ is the set of all possible annotation sequences of sentence *X*.

The negative log-likelihood is used to estimate the training, and the training target can be expressed as

(18) $$\begin{array}{c} L\left(\theta \right)=-\frac{1}{\left|\delta \right|}\sum_{\left(X,y\right)\in \delta }\log\left[p\left(y|X,\theta \right)\right]\\ =\frac{1}{\left|\delta \right|}\sum_{\left(X,y\right)\in \delta }\left[\log\left(\sum_{\tilde{y}\in Y_{X}}e^{s\left(X,\tilde{y},\theta \right)}\right)+s\left(X,y,\theta \right)\right]. \end{array}$$

*δ* is the training sample set.

In the decoding process, the dynamic programming algorithm is used to calculate the score of the sentence that finally selects the labeling sequence. The sequence with the highest score can be expressed as

(19) $$\begin{array}{c} y^{*}=\arg\underset{\tilde{y}\in Y_{X}}{\max}s\left(X,\tilde{y}\right). \end{array}$$

Maximum separation method: assuming that *x*^(*i*)^ is a given sample and *y*^(*i*)^ is a correct category, then the training set *S* can be expressed as

(20) $$\begin{array}{c} S=\left\{\left(x^{\left(1\right)},y^{\left(1\right)}\right),\left(x^{\left(2\right)},y^{\left(2\right)}\right),\ldots ,\left(x^{\left(n\right)},y^{\left(n\right)}\right)\right\}. \end{array}$$

According to the model prediction, the category can be obtained as shown in equation (21) as follows:

(21) $$\begin{array}{c} h\left(x^{\left(i\right)}\right)=\arg\underset{y:g\left(x,y\right)\leq 0}{\max}W^{T}f\left(x,y\right). \end{array}$$

*f*(*x*, *y*) is the characteristic function, and *g*(*x*, *y*) is the model restriction condition. It is necessary to establish a loss function to measure the model's performance. Suppose that the maximum interval method calculates the distance between the real category *y*^(*i*)^ and the predicted category *h*(*x*^(*i*)^), which is reduced during the training process and used as part of the loss function. The loss function of the *i*-th sample is established as shown in

(22) $$\begin{array}{c} l_{i}\left(w\right)=\underset{\hat{y}\in GEN\left(x^{\left(i\right)}\right)}{\max}\left(w^{T}f\left(x,\hat{y}\right)+\Delta -w^{T}f\left(x,y^{\left(i\right)}\right)\right). \end{array}$$

*GEN*(*x*^(*i*)^) is a given sample *x*^(*i*)^ to produce all possible prediction results.

The maximum interval loss function for the model is established, let $\Delta \left(y^{\left(i\right)},\hat{y}\right)$ be the structured interval loss, *y*^(*i*)^ is the correct label sequence of the *i*-th sample, and $\hat{y}$ is the sequence predicted by the model. The loss function is

(23) $$\begin{array}{c} \Delta \left(y^{\left(i\right)},\hat{y}\right)=\sum_{t=1}^{m}\mu \left\{y^{\left(i\right),t}\neq {\hat{y}}^{t}\right\}. \end{array}$$

*μ* is the attenuation parameter, and *m* is the character length of the sample sentence *x*^(*i*)^. When a training set is given as *ξ*, the objective loss function added by *l*_2_ norm is expressed as

(24) $$\begin{array}{c} L\left(\theta \right)=-\frac{1}{\left|\xi \right|}\sum_{\left(x^{\left(i\right)},y^{\left(i\right)}\right)\in \xi }l_{i}\left(\theta \right)+\frac{\lambda }{2}{\left\|\theta \right\|}_{2}^{2}. \end{array}$$

(25) $$\begin{array}{c} l_{i}\left(\theta \right)=\underset{\hat{y}\in GEN\left(x^{\left(i\right)}\right)}{\max}\left[s\left(x^{\left(i\right)},\hat{y},\theta \right)+\Delta \left(y^{\left(i\right)},\hat{y}\right)-s\left(x^{\left(i\right)},y^{\left(i\right)},\theta \right)\right]. \end{array}$$

*θ* represents the model parameters, *GEN*(*x*^(*i*)^) is all possible prediction results produced by a given sample *x*^(*i*)^, and $\Delta \left(y^{\left(i\right)},\hat{y}\right)$ is the structured interval loss.

### 3.5. Establishment of the Bi-LSTM-CRF Model

The three named entities of person, place, and organization in the legal text are identified. The specific experimental process is shown in Figure 4.

The Bi-LSTM-CRF model can be divided into the Bi-LSTM layer and the CRF layer. The function of the Bi-LSTM layer is to extract contextual information through the input words and word vectors and determine the probability of a certain type of label making the prediction. The CRF layer is used to consider the correlation between tags. The Bi-LSTM-CRF model structure is shown in Figure 5.

### 3.6. Data Source and Parameter Setting

The data set is used from the exercise contest folder in “China AI and Law Challenge” CAIL2018_ALL_DATA.zip. There are 154,592 training sets, 32,508 test sets, and 17,131 verification sets, with 204,231 data in the folder. The data in the exercise_contest file are programmed to extract the text content to form the CLNER data set. The legal documents used are sensitively processed data, containing many names of individuals, places, and organizations, and the text has a high density of entities. The data used in this paper are the Marked_Fact data set, which is processed by word segmentation. BIO annotation is used to obtain annotated corpus and divide the corpus into the training set and test set. The python version used in the experiment is 3.6. The TensorFlow version is 1.13.1. The parameters of Bi-LSTM-CRF model training are set as follows: dropout means that during the training process of the DNN, the neural network unit temporarily discards it from the network according to a certain probability. Dropout can prevent overfitting. The dropout parameter value is 0.5, Word2Vec word vector dimension value is 300, and the hidden layer dimension parameter value is 300. The learning rate is an essential hyperparameter in deep learning, determining whether the objective function can converge to a local minimum and when it converges to the minimum. A reasonable learning rate can make the objective function link to a local minimum in an adequate time. The learning rate is 0.001. The optimizer is Adam. The Epoch parameter is 15. The batch parameter is 64.

## 4. Results and Discussion

### 4.1. Analysis of Bi-LSTM-CRF Model Recognition Results Using Different Annotation Methods

The recognition result of the Bi-LSTM-CRF model is shown in Figure 6.

Figure 6 shows that the accuracy rate on the named entity is 86.54%, the recall rate is 87.86%, and the F1 value is 87.20%. The accuracy rate on the place name entity is 68.09%, the recall rate is 67.12%, and the F1 value is 67.60%. The accuracy rate on the named entity is 89.91%, the recall rate is 88.98%, and the F1 value is 89.45%. The model trained on the word sequence labeling corpus was found to have an immense F1 value on the two types of entities: person name and organization name.

Using the labeling method of character segmentation and using characters as the input of the model, the recognition result of the Bi-LSTM-CRF model is shown in Figure 7.

Figure 7 shows that the accuracy rate on the named entity is 87.06%, the recall rate is 89.23%, and the F1 value is 88.13%. The accuracy rate on the place name entity is 68.92%, the recall rate is 65.67%, and the F1 value is 67.26%. The accuracy rate on the named entity is 84.65%, the recall rate is 82.81%, and the F1 value is 83.72%. The model trained on the word sequence labeling corpus can obtain an immense F1 value on the two types of entities, the name of the person and the name of the organization.

The model recognition results of the labeling methods are compared using character segmentation and word segmentation, as shown in Figure 8.

Figure 8 shows that the F1 value obtained by the model trained on a single character sequence labeling corpus is higher than that of the two or more character sequence labeling corpus and for the two types of entities: place name and organization name. The F1 value obtained by the Bi-LSTM-CRF model using segmentation of two or more words will be higher. Therefore, through comparison, the Bi-LSTM-CRF model using segmentation of two or more words is more suitable for length recognition of more extended entities.

### 4.2. Analysis of Bi-LSTM-CRF Model Recognition Results Using Different Objective Loss Functions

The results of parameter learning using log-likelihood are shown in Figure 9.

Figure 9 shows that the accuracy rate on the named entity is 79.2%, the recall rate is 83.03%, and the F1 value is 81.07%. The accuracy rate on the place name entity is 66.25%, the recall rate is 65.12%, and the F1 value is 65.7%. The accuracy rate on the named entity is 82.91%, the recall rate is 83.98%, and the F1 value is 83.4%.

The result of parameter learning using the maximum interval criterion is shown in Figure 10.

Figure 10 shows that the accuracy rate on the named entity is 79.17%, the recall rate is 82.97%, and the F1 value is 81.03%. The accuracy rate on the place name entity is 66.13%, the recall rate is 65.03%, and the F1 value is 65.58%. The accuracy rate on the named entity is 82.78%, the recall rate is 83.69%, and the F1 value is 83.23%. The model trained using the parameter learning of the maximum interval criterion obtains the enormous F1 value on the entity name.

The F1 values are compared using different objective loss functions, as shown in Figure 11.

Figure 11 shows that the F1 value of parameter learning using log-likelihood is larger than the F1 value using different objective loss functions. This result appears because the maximum interval method is a nonprobabilistic model, and the loss is the signal distance between the actual model and the hypothetical model. The likelihood estimation method is a probability model. Its log loss measures the difference between the accurate conditional probability distribution and the theoretical conditional probability distribution. The Bi-LSTM model is used to obtain character information features, while the CRF model marks the character assignment, a dependent probability model. Therefore, the log-likelihood parameter learning result is better than the parameter learning result using the maximum interval criterion. Therefore, the likelihood estimation method is more suitable for the Bi-LSTM-CRF model than the complete interval method.

Although the context information output by the Bi-LSTM layer can also get the NER result through the softmax layer, the result obtained directly through the Bi-LSTM layer only considers the context information. The output result of the Bi-LSTM layer does not take into account the dependencies between tags. The CRF model can learn some global-based constraint information through corpus training to consider the dependency relationship between markers. Therefore, the Bi-LSTM-CRF model is adopted. This model can use the Bi-LSTM layer to extract the context information of the text to predict the label and add some constraint rules through the CRF layer to ensure that the final recognition result is reasonable. Through the introduction of related theories and experimental results, the legally NER method based on the character-level neural network has the following advantages: (1) compared with the traditional method, the method based on deep learning avoids the design of artificial feature engineering and solves the dimensional disaster problem caused by the sparse data in the traditional method; (2) the model uses the Bi-LSTM-CRF model to obtain contextual information, which solves the long-distance dependence problem of ordinary models.

## 5. Conclusions

With the rapid development of AI technology, deep learning models have been increasingly widely used in the judicial field, especially the application of deep learning models to NER in legal texts. Since there are few studies on NER at present, this paper studies NER in legal texts using deep learning models. First, the Bi-LSTM-CRF model is established. Then, it sets different objective loss functions and uses other labeling methods to compare and analyze the entity recognition effects of the established models. The research results show that the F1 value obtained by the model trained through the word sequence labeling corpus on the person's name entity is higher than that of the word sequence labeling corpus. The F1 value obtained by the Bi-LSTM-CRF model using word segmentation will be higher for the two types of entities, place names and organization names. The Bi-LSTM-CRF model using word segmentation is more suitable for recognizing more extended entities. The parameter learning result using log-likelihood is better than the parameter learning result using the maximum interval criterion, and it is more suitable for the Bi-LSTM-CRF model. This paper provides ideas for the research of legal text recognition and has a particular value. The disadvantage of this paper is that it only recognizes three types of entities in the legal text, names of persons, names of places, and names of organizations. However, there are many entities in the legal text, so the legal text's crimes, legal provisions, and other entities can be studied later. In the future, more entity types will be trained and labeled by the model. As a result, more entities in the legal text will be identified.

## Figures and Tables

**Figure 1:** The judgment criteria of NER.

**Figure 2:** LSTM network structure.

**Figure 3:** The process of LSTM network model training.

**Figure 4:** Flow chart of NER experiment.

**Figure 5:** Bi-LSTM-CRF model structure.

**Figure 6:** Bi-LSTM-CRF model recognition results using word segmentation.

**Figure 7:** Bi-LSTM-CRF model recognition results using character segmentation.

**Figure 8:** Comparison of model recognition results using different annotation methods.

**Figure 9:** Parameter learning results using log-likelihood.

**Figure 10:** Parameter learning using the maximum interval criterion.

**Figure 11:** Comparison of F1 values using different objective loss functions.

**Table 1:** Standard name combining the BIO labeling method and entity labeling method.

Entity category	Start tag	Middle-end tag
PER	B-PER	I-PER
LOC	B-LOC	I-LOC
ORG	B-ORG	I-ORG

## Data Availability

The data used to support the findings of this study are included in the article.
